# Design and Workspace Analysis of a Parallel Ankle Rehabilitation Robot (PARR)

This article has been retracted.

**DOI:** 10.1155/2019/4164790

**Published:** 2019-03-14

**Authors:** Leiyu Zhang, Jianfeng Li, Mingjie Dong, Bin Fang, Ying Cui, Shiping Zuo, Kai Zhang

**Affiliations:** ^1^College of Mechanical Engineering and Applied Electronics Technology, Beijing University of Technology, Beijing, China; ^2^Department of Computer Science and Technology, Tsinghua University, Beijing, China; ^3^Department of Gynaecology and Obstetrics, China-Janpan Friendship Hospital, Beijing, China

## Abstract

The ankle rehabilitation robot is essential equipment for patients with foot drop and talipes valgus to make up deficiencies of the manual rehabilitation training and reduce the workload of rehabilitation physicians. A parallel ankle rehabilitation robot (PARR) was developed which had three rotational degrees of freedom around a virtual stationary center for the ankle joint. The center of the ankle should be coincided with the virtual stationary center during the rehabilitation process. Meanwhile, a complete information acquisition system was constructed to improve the human-machine interactivity among the robot, patients, and physicians. The physiological motion space (PMS) of ankle joint in the autonomous and boundary elliptical movements was obtained with the help of the RRR branch and absolute encoders. The natural extreme postures of the ankle complex are the superposition of the three typical movements at the boundary motions. Based on the kinematic model of PARR, the theoretical workspace (TWS) of the parallel mechanism was acquired using the limit boundary searching method and could encircle PMS completely. However, the effective workspace (EWS) was smaller than TWS due to the physical structure, volume, and interference of mechanical elements. In addition, EWS has more clinical significance for the ankle rehabilitation. The PARR prototype satisfies all single-axis rehabilitations of the ankle and can cover most compound motions of the ankle. The goodness of fit of PMS can reach 93.5%. Hence, the developed PARR can be applied to the ankle rehabilitation widely.

## 1. Introduction

With the increasing incidence of stroke and frequent traffic accidents, a high proportion of patients have lower limb motor dysfunction due to foot drop or ankle joint injuries. In addition, the clubfoot and valgus are common causes of orthopedics in teenagers and children. It is necessary to perform the ankle dissection and orthopedic surgery to improve the lower extremity motor function and gait reconstruction. The above patients need to carry out extensive and repetitive rehabilitation training for the ankle joint. Traditional rehabilitation training is a one-on-one manual treatment for patients. The disadvantages are inefficiency, high labor intensity, and lack of scientific and effective data monitoring and feedback. It is difficult to numerically evaluate the patient's rehabilitation status. Parallel robots with high stiffness allow for various treatment modes and the real-time information collection, such as adaptive training and highly repetitive movements.

Throughout the past few decades, various parallel robots, due to their large payload capacity, high stiffness, and accuracy in a safe workspace [1], have been widely developed for ankle rehabilitation. The most popular instance is the Rutgers Ankle proposed by Girone et al. [2], which is a pneumatically actuated parallel robot with six degrees of freedom (6-DOFs). The Rutgers Ankle allows patients to receive treatment in a virtual reality environment and has been successfully used on patients with stroke sequelae and musculoskeletal injuries. Subsequently, to better align the number of the robot's DOFs with that of the ankle complex, studies were performed to focus on lower-mobility parallel robots. Dai et al. [3] presented a mechanism synthesis technique based on an ankle orientation presentation and then developed several 3-DOFs and 4-DOFs parallel mechanisms with a central strut. According to the movement analysis of the ankle, Liu et al. [4] put forth a 3-RSS/S parallel mechanism with a compact structure, low inertia, and comparatively good carrying capacity, where R and S denoted the rotational joint and the spherical joint, respectively. Saglia et al. [5] proposed a redundantly actuated parallel robot for the plantarflexion/dorsiflexion and inversion/eversion of the ankle joint, in which a fairly simple kinematic configuration (i.e., 3-UPS/U parallel mechanism, U and P denoted the universal joint, and the prismatic joint) was adopted as the main mechanical structure. Notably, stemming from the utilization of a central strut, the rotation center of the moving platform in these three studies was misaligned with that of the ankle (i.e., the robot did not remain compatible with the ankle), leading to inconveniences for patients (i.e., patients were required to shift their sitting postures repeatedly during the rehabilitation process) due to large changes in the ankle position and coupled motions of the shank and the foot [6]. Tsoi et al. [7] presented an approach to achieving an aligned rotation center by utilizing the ankle as a part of the robot kinematic constraint, including selecting four linear actuators to produce obliquity of the moving platform. Since the calves and ankle joint should be kept as stationary as possible during the rehabilitation process, safety issues caused by unexpected excessive loads cannot be ignored. Thus, these study results indicate that compatibility, convenience, and safety issues should be considered in the design process.

Jamwal et al. [8] proposed a light weight and compliant parallel ankle rehabilitation robot by placing pneumatic muscle actuators (PMAs) parallel to the patient's shinbone. Due to the skeletal muscle-like behavior and anatomically correct arrangement of PMAs, the robot remains compatible with the ankle during different treatment modes. Moreover, three physical rotation axes were set to address the safety issues [9]. A fuzzy controller was developed to compensate for the nonlinear and transient nature of PMAs. Subsequently, to enhance patients' cooperation during the rehabilitation process, an interactive training paradigm based on impedance control was developed and evaluated [1, 10]. Several multiobjective optimization schemes [11–14] were also carried out to provide better design solutions. Two kinds of serial spherical mechanisms, also called equivalent spherical joints, with a symmetrical structure were designed by Wang et al. [15] to actualize 3-DOFs rotational motion and ensure the mechanism center of rotation matches that of the ankle. Three types of 3-UPS/RRR redundantly actuated parallel mechanisms were selected to analyze and compare their kinematic performance, in which the redundant actuator was installed on the serial spherical mechanism to achieve the features of no singularity, better dexterity, and higher stiffness. Analogous to study [15], a 3-RUS/RRR redundantly actuated parallel mechanism was designed and analyzed by Wang et al. [16], the prototype of which was built according to geometrical parameters selected via multiobjective optimization [17]. Zhang et al. [9] presented a redundantly actuated reconfiguration robotic design called CARR, which was driven by four Festo fluidic muscles; and the robot provided an adjustable workspace and actuator torque to meet the requirements of range of motion exercises and muscle strengthening exercises. Subsequently, a trajectory tracking controller was implemented on the prototype of CARR [18], and the potential for clinical application was supported via a preliminary study. Although actuator redundancy is a common approach to improving robot's kinematic performance and avoiding singularity configuration [7–18], it may complicate the structure and control scheme.

Based on the above research and analysis, a 2-UPS/RRR configuration is selected and a parallel ankle rehabilitation robot (PARR) with two UPS branches and three rotational joints is developed taking physical properties of the ankle joint into consideration, where P and R denotes the active prismatic and rotational joints, respectively. The rotation center should coincide with that of ankle joint approximately when the patient puts the affected foot onto the upper platform of PARR. The theoretical workspace (TWS) of PARR can be obtained by solving the inverse solution of the mechanism and establishing the corresponding Jacobian matrix. The physiological motion space (PMS) of the ankle joint is measured by means of the three rotational DOFs of the rehabilitation robot when the two branches are disassembled at the upper ends. In order to evaluate the kinematic performance and actual workspace of PARR, the effective workspace (EWS) can be measured and acquired during the autonomous movements at the largest possible range. EWS, which is an important indicator of a parallel robot, directly affects the therapeutic schedules made by physical therapists and the expected recoveries of patients. Hence, EWS has more clinical significance for the ankle rehabilitation. Furthermore, the goodness of fit of the human-machine system is analyzed through comparing the three ranges of motion mentioned above.

## 2. Design of Ankle Rehabilitation Robot

The ankle includes three joints: the ankle joint or talocrural joint, the subtalar joint, and the inferior tibiofibular joint [19]. The bony architecture of the ankle consists of three bones: the tibia, the fibula, and the talus. The movements produced at the ankle are plantarflexion/dorsiflexion (PL/DO) of the foot mainly. The other movements, adduction/abduction (AD/AB) and inversion/eversion (IN/EV), can keep human bodies balanced and assist walking steering during the walking and standing positions [20]. Hence, the ankle joint can be simplified as a spherical joint [21, 22] with three rotational DOFs described as rotating around *x*_an_, *y*_an_, and *z*_an_ axes at the coordinate system {*o*_an_}, as shown in Figure 1.

For the ankle rehabilitation, the configuration of parallel robot should possess 3-DOFs rotational motion and sufficient range of motion (ROM). A configuration without redundant branches is selected by the method of the topological analysis and configuration optimization. A 2-UPS/RRR parallel ankle rehabilitation robot (PARR) was developed which had three rotational DOFs around a virtual stationary center for the ankle joint. It consists of a constrained branch and two drive ones, as shown in Figure 2. The constrained one with the configuration RRR is composed of three rotational joints, denoted by R_1_, R_2_, and R_3_, respectively, which are connected in series. The joint R_1_ is installed vertically and used as an active joint. In addition, the three axes are perpendicular to each other and intersected at the origin *o*_0_ of the coordinate system {0} (Figure 3). The configuration UPS is selected as the drive branch and the joint P is used as the active joint to simplify the structure of the driven units.

The detailed structure of the rehabilitation robot is shown in Figure 2. Two identical linear actuators are employed as the active joint P_1_ and P_2_ in the two UPS branches, and the stepper motor drives the joint R_1_ via a planetary reducer (reduction ratio 12 : 1). In order to monitor the angles and angular velocities of the constrained branch RRR in real time, three absolute encoders are installed at each rotational joint. The encoder 1# measures the kinematics information of R_1_ by means of gear meshing. The encoders 2# and 3# are directly connected in series with the rotating shafts of R_2_ and R_3_, respectively. By acquiring the angles of the encoders, the accurate attitude of the moving platform can be obtained timely. The control system regulates the movement speeds of linear actuators and the stepping motor, realizes the closed loop motion control of PARR based on the collected kinematic information.

The moving platform composed of upper and lower platforms is connected to joints R_3_, S_1_, and S_2_ simultaneously, as shown in Figure 4. The patient puts the affected foot onto the upper platform. The heel abuts the baffle and adjusts its anteroposterior position where the baffle's position can be changed according to the foot's size. Meanwhile, the foot position in the height direction can be changed by increasing or decreasing the number of customized insoles fixed on the upper platform. The customized insoles have three specifications with different thicknesses (e.g., 1 mm, 2 mm, and 3 mm), and the ideal height of the affected foot can be acquired by the combination of different specifications. The therapist adjusts the position and attitude of the foot and can keep the misalignments between the rotation centers of the human-machine system within 2 mm. In addition, the elastic straps are used to tie the affected foot on the upper platform to avoid large misalignments and maintain sufficient connection strength. Four force sensors and a torque sensor (Green color) are added to the moving platform. The active forces applied on the platform during the movements of PL/DO and IN/EV can be measured by the four force sensors. The motion intention of patients is estimated and predicted according to the force distribution. In order to detect the torques of AD/AB, a torque sensor (M2210G, SRI Inc., China) is connected and installed perpendicular to the platform. Hence, the force/torque sensors and the absolute encoders constitute a complete information acquisition system to measure the kinematic and dynamic information of PARR. The velocity measurements of the encoders are usually used to compensate kinetic friction. The breakaway friction can be compensated with the use of the additional force/torque sensors that directly measures the interaction force between the human and the robot. Hence, the stepper motor and linear actuators are backdrivable during the human-interaction training, and the robot can easily be moved manually by a therapist in order to release the patient from a potentially uncomfortable posture.

Before finalizing the detailed structure of PARR, the relevant kinematic analysis performed in Section 3 and Section 4 is quite essential to determine the dimensions of key components and main technical specifications of drive elements, especially the moving range of linear actuators, distribution of the sensors, theoretical workspace, etc. A PARR prototype was developed based on the detailed structure, and the aluminum alloy 7075 was widely used in structural parts to ensure the sufficient strength and light weight, as shown in Figure 5. In addition, the device capabilities are provided in Table 1.

PARR possesses three training modes: passive mode, active mode, and human-interaction mode. Patients can select suitable modes according to the muscle strength grade of ankle joint. During the uniaxis or multiaxis passive training process, the ankle joint is driven along the recovery trajectory planned by physical therapists. When the ankle joint has sufficient strength to exercise, the active mode can be adopted. The rehabilitation robot detects the motion intention of the patient based on the force/torque imposed by the sole and the ankle joint and assists the ankle joint to move according to the patient's motivation. With the accumulation of rehabilitation effect, the human-machine interaction mode will be employed to train the muscle strength and ROM of the ankle joint. The motion impedance of PARR can be changed through controlling the force/torque of the moving platform. Through establishing a complete kinematic information acquisition system, the interaction force/torque and the path trajectory during the different training movements are measured and recorded. In addition, the path recording function can be used to replicate the rehabilitation path when a physical therapist moves the platform along a customized trajectory. Hence, the interactions between the robot, patients, and therapists are improved. The physical therapists can perform real-time observations and evaluations of the rehabilitation process based on the collected data and quantitatively analyze the rehabilitation effect of the ankle complex.

## 3. Kinematic Analysis of PARR

The kinematic analysis of the rehabilitation mechanism is of great significance for workspace analysis, motion trajectory planning, and performance analysis. Therefore, it is necessary to establish kinematic model to analyze the relevant kinematics of PARR.

Several coordinate systems should be built on the rehabilitation mechanism to establish the kinematic model, as shown in Figure 3. A static coordinate {0} is fixed at the virtual stationary center of PARR where the original point is denoted by *o*_0_ and the axes *x*_0_, *y*_0_, and *z*_0_ are parallel to those of joints R_2_, R_3_, and R_1_ at the initial position, respectively. A moving coordinate {4} is fixed on the moving platform and moved together. The two coordinates {0} and {4} are coincident at the initial position as shown in Figure 3. The first and second axis of the universal joint U_*i*_ (*i* = 1, 2), denoted by *u*_1,*i*_ and *u*_2,*i*_, are parallel to *x*_0_ and *y*_0_. In order to make the coordinate systems clearer, the coordinate systems are placed beside the schematic diagram and connected by imaginary lines. The coordinate {1, *i*} is built on the geometric center *a*_*i*_ of U_*i*_, and the axis *x*_1,*i*_ is arranged along *u*_1,*i*_. Similarly, another axis *y*_1,*i*_ is parallel to *u*_2,*i*_ at the initial position. The coordinate {2, *i*} is also established on the center *a*_*i*_ of U_*i*_ which is the virtual intersection point of joints P_*i*_ and U_*i*_. The axes *y*_2,*i*_ and *z*_2,*i*_ are parallel to *u*_2,*i*_ and the axis of joint P_*i*_, separately. A coordinate {3, *i*} is built at the center *c*_*i*_ of the spherical joint S_*i*_, and the three axes are parallel to those of {2, *i*} at the initial position.

Since PARR always rotates around the stationary point *o*_0_, it is convenient to employ the *Z*-*X*-*Y* Euler angle to describe the attitude angles of the moving platform. The symbols *α*, *β*, and *γ* denote the angles of PL/DO, IN/EV, and AD/AB, respectively. The three Euler angles also represent the angles rotating around the axes *x*_0_, *y*_0_, and *z*_0_. When *α*, *β*, and *γ* are known, the rotation transformation matrix of the moving coordinate system {4} with respect to the fixed coordinate system {0} can be expressed as

(1) R40=Rzγ·Rxα·Ryβ.

Given the attitude angles *α*, *β*, and *γ* of the moving platform, the inverse kinematics method is applied to solve the inputs of linear actuators (in joints P_1_ and P_2_) and the stepper motor (in the joint R_1_). The closed vector loop of the drive branch U_*i*_P_*i*_S_*i*_ is constructed, as shown in Figure 6. The position vector ^0^***r***_*c*,*i*_ of the geometric center *c*_*i*_ of joint S_*i*_ in the coordinate {0} is given by

(2) r0c,i=r0o,4+R40×r4c,i,

(3) r0c,i=r0a,i+l2,i·z2,i=r0a,i+l2,i·R20·001,

where, ^0^***r***_*a,i*_, ^0^***r***_*c,i*_, and ^0^***r***_*o,*4_ denote the vectors of points *a*_*i*_, *c*_*i*_, and *o*_4_ in the coordinate {0}; *l*_2,*i*_ denotes the length of segment *a*_*i*_*c*_*i*_ and the linear actuator; ^4^***r***_*c,i*_ is the position vector of point *c*_*i*_ in the coordinate {4}; _2_^0^**R** denotes the rotation transformation matrix of the coordinate {2} with respect to {0} and can be calculated by

(4) R20i=R10i·R21i,R21i=cθ2,i0sθ2,isθ1,i·sθ2,icθ1,i−cθ2,i·sθ1,i−cθ1,i·sθ2,isθ1,icθ1,i·cθ2,i,

where *θ*_1,*i*_ and *θ*_2,*i*_ denote the rotation angles of U_*i*_ around the axes *u*_1,*i*_ and *u*_2,*i*_; *c* and *s* are abbreviations of cos and sin, respectively.

Combining equations (2) and (3), we can get

(5) l2,i=r00,4+40R·r0c,i−r0a,i.

The rotation angle *θ*_3_ of the active joint R_1_ is equal to the Euler angle *γ*, where

(6) $$\begin{array}{c} \theta_{3}=\gamma . \end{array}$$

The inputs *l*_2,1_, *l*_2,2_, and *θ*_3_ can be obtained by solving equations (5) and (6).

## 4. Workspace Analysis of PARR

EWS is an important indicator to evaluate the kinematic performance of a robot, which directly affects the practical application value. EWS of this parallel robot is the reachable workspace of the PARR prototype through taking the parts sizes and interferences into consideration. To determine whether PARR can meet the space requirement, it is necessary to measure PMS of the ankle joint in the global movements.

### 4.1. PMS of Ankle Joint

The literature [23] measured ROM of the ankle joint during the three uniaxial motions. PMS of the ankle in the global motion range still has insufficient description and data. In order to better evaluate the fit of the human-machine motion space, a test and experimental platform was designed to measure PMS during a full range of the ankle's autonomous motion.

The experimental platform was constructed conveniently by removing the two UPS branches and the stepper motor of R_1_. Only the RRR branch which consisted of three passive joint R was retained, as shown in Figure 7(a). In addition, the RRR branch itself had enough motion range for the ankle after the relevant parts were removed. The absolute encodes mentioned above were applied to measure the angles of three R joints (Figure 2). In order to reduce the influences of the thigh and calves on the movements of the ankle joint, they were tied and fixed with wooden clamps and elastic straps, as shown in Figure 7(b). In the initial position, the thigh, sole, and moving platform approximately remained parallel and level. The participant's foot was tied to the platform using straps, as shown in Figure 7(c), ensuring adequate connection strength and force transmission performance. The center of ankle joint should be approximately coincident to the virtual stationary center of PARR through adjusting the baffle position and the number of insoles.

In the measurement experiments, the ankle completed a full range of autonomous motion and a boundary elliptical motion. During the autonomous motions, the participants maximally moved the right or left ankle to do PL/DO and IN/EV at all different adduction/abduction planes. The boundary elliptical motion was a compound motion of the three movements along the physiological movement boundary. A group of fifteen healthy Chinese individuals were enrolled in this experiment. The participants consisted of nine males (average age = 26, average height = 175.5 cm, and average weight = 68.5 kg) and six females (average age = 25, average height = 162.5 cm, and average weight = 55.5 kg). All measurement sessions consisted of a sequence of motor tasks followed by a short resting phase. Participants performed 5 to 7 exercise cycles lasting 30 seconds each, followed by a 2-minute resting period (total time for each session, 4–6 min).

PMS of the ankle joint in the autonomous movements was obtained through recording all the angle data in a space rectangular coordinate system, as shown in Figure 8. The angle data used in PMS were the mean value of the fifteen participants. The shape of PMS was almost like a cube, and each surface bulged outward at the middle. ROM of the ankle joint reached the maximum at the initial position (*α* = *γ* *=* *β* = 0°) and descended with the increase or decrease of any attitude angle. For further analysis of PMS, it was projected on the three plane of the coordinate system {*o*_an_}, as shown in Figure 9. The PL/DO movements are the most important during the walking. The AD/AB angle *γ*_PMS_ of the ankle joint had little influence on the motion range of the PL/DO angle *α*_PMS_. In addition, the range of *γ*_PMS_ shrank asymmetrically with the IN/EV angle *β*_PMS_.

The boundary elliptical motion is that the ankle tries to rotate along the maximum boundary, and the tiptoe draws an ellipse gently. The three attitude angles of all limit postures are depicted in Figure 10. The angle *α*_PMS_ varied periodically and sinusoidally with the time; the angles *γ*_PMS_ and *β*_PMS_ changed along a cosine shape. ROM in the boundary motions was consistent with that of autonomous movements. Furthermore, we could find that the natural extreme postures of the ankle complex were the superposition of the three typical movements. Hence, it is necessary to exercise the compound motions of the ankle complex.

### 4.2. Workspace of PARR

TWS is defined as a set of all postures without regard to interferences among different parts and drive units. The theoretical sizes or coordinates of points are listed in Table 2. Based on the kinematic model of PARR in Section 2, TWS of the parallel mechanism can be solved and acquired using the limit boundary searching method, as shown in Figure 11. Compared with PMS of the ankle joint, TWS is a larger cube and can encircle PMS completely. The ranges of uniaxial movements are enough for the ankle complex: −46.2° < *α*_TWS_ < 30°, −23.5° < *β*_TWS_ < 23.5°, −36° < *γ*_TWS_ < 36°, where *α*_TWS_, *β*_TWS_, and *γ*_TWS_ denote the attitude angles of joints R_2_, R_3_, and R_1_ (Figure 5), respectively.

The effective workspace (EWS) of PARR was acquired by measuring the movements of R_1_, R_2_, and R_3_ during the autonomic movements. A measuring program was made for the autonomic movements to control the prototype and detect the angles of the three rotational joints. Firstly, the angle of R_1_ in the PARR prototype, denoted by *γ*_EWS_, was measured through driving the prototype from the left to the right extreme position. Then, the corresponding angles of R_2_ and R_3_, denoted by *α*_EWS_ and *β*_EWS_, were measured and recorded separately with a 2° interval of *γ*_EWS_. EWS of the PARR prototype was obtained when the prototype traversed all reachable workspace (Figure 11). EWS is smaller than TWS due to the physical structure, volume, and interference of mechanical elements. However, EWS has more clinical significance and practical application value for the ankle rehabilitation.

Based on the above results, both PMS and EWS are put into a space rectangular coordinate system to analyze the goodness of fit of the human-machine system, as shown in Figure 12. It can be found that the two workspaces possess high goodness of fit and PARR can almost meet all the physiological movements of the ankle. The goodness of fit *η* of PMS is calculated by

(7) $$\begin{array}{c} \eta =\frac{V_{\text{overlap}}}{V_{\text{PMS}}}\times 100\%\\ =93.5\%, \end{array}$$

where *V*_overlap_ is the overlap volume of PMS and EWS and *V*_PMS_ denotes the volume of PMS.

For further analysis of the goodness of fit, PMS and EWS are projected on the three planes of the coordinate {0}, as shown in Figure 13. The PARR prototype nearly satisfies all uniaxis rehabilitations of the ankle, and the relevant technical parameters are listed in Table 3. In addition, PARR can meet the rehabilitations of PL/DO and IN/EV movements at any AD/AB angle *γ*_EWS_. The range of *α*_EWS_ shrinks symmetrically with the angle *β*_EWS_, as shown in Figure 13(a). Hence, the motion range of PL/DO movements will be reduced slightly when the ankle joint remains a large IN/EV angle.

## 5. Conclusions

For the extensive and repetitive rehabilitation training for the ankle joint, a PARR prototype with the 2-UPS/RRR configuration was developed which had three rotational degrees of freedom around a virtual stationary center. PARR possessed the advantage of compact structure, excellent human-machine compatibility, and higher effective workspace. A complete information acquisition system was constructed to measure and record the interaction force/torque and the path trajectory during the rehabilitation movements. The interactions between the robot, patients, and therapists could be promoted greatly. PMS of ankle joint in the autonomous and boundary elliptical movements was obtained with the help of the RRR branch and absolute encoders. The natural extreme postures of the ankle complex are the superposition of the three typical movements at the boundary motions. The conventional uniaxial trainings cannot meet the requirements of ankle rehabilitation. It is necessary to exercise the compound motions of the ankle. Based on the kinematic model of PARR, TWS of the parallel mechanism was acquired by use of the limit boundary searching method and can encircle PMS completely. Furthermore, EWS, which had more clinical significance, was acquired by measuring the movements of R_1_, R_2_, and R_3_ during the autonomic movements. EWS is smaller than TWS due to the physical structure, volume, and interference of mechanical elements. The PARR prototype satisfies all single-axis rehabilitations of the ankle and can cover most compound motions of the ankle. In addition, the goodness of fit of PMS can reach 93.5%. Hence, the developed PARR may be applied to the ankle rehabilitation widely.

## Figures and Tables

**Figure 1:** Skeletal structure of the ankle joint.

**Figure 2:** Structure of PARR.

**Figure 3:** Schematic diagram of PARR.

**Figure 4:** Structure of the moving platform.

**Figure 5:** PARR prototype.

**Figure 6:** Closed vector loop of U_*i*_P_*i*_S_*i*_.

**Figure 7:** Measurement experiments of PMS. (a) RRR branch of PARR. (b) Wooden clamp. (c) Experimental platform.

**Figure 8:** PMS of ankle joint.

**Figure 9:** Projections of PMS at the coordinate {*o*_an_}. (a) Plane *x*_an_*o*_an_*y*_an_. (b) Plane *y*_an_*o*_an_*z*_an_. (c) Plane *x*_an_*o*_an_*z*_an_.

**Figure 10:** Attitude angles in the boundary elliptical motion.

**Figure 11:** TWS and EWS of PARR.

**Figure 12:** PMS and EWS.

**Figure 13:** Projections of PMS and EWS at the coordinate {*o*_0_}. (a) Plane *x*_0_*o*_0_*y*_0_. (b) Plane *y*_0_*o*_0_*z*_0_. (c) Plane *x*_0_*o*_0_*z*_0_.

**Table 1:** Device capabilities of PARR.

Volume (mm)	Weight (kg)	Height of upper platform (mm)	Max. continuous torque (N · *m*)		
			PL/DO	AD/AB	IN/EV
430 ∗ 400 ∗ 460	15.6	326	65.2	20.6	63.9

**Table 2:** Theoretical parameters of PARR.

Parameters	Value (mm)	Parameters	Value (mm)
*l*_1,*i*_	192	*o*_0_	(0, 0, 0)
*l*_2,*i*_	255 ≤ *l*_2,*i*_ ≤ 405	*c*_1_	(130, 129.5, −12.5)
*l*_0_	421	*c*_2_	(−130, 129.5, −12.5)
*θ*_1,*i*_	−35° ≤ *θ*_1,*i*_ ≤ 35°	*a*_1_	(175, 80, −421)
*θ*_2,*i*_	−35° ≤ *θ*_2,*i*_ ≤ 35°	*a*_2_	(−175, 80, −421)

**Table 3:** Single motion ranges of ankle joint and PARR.

Motion type	Ankle joint	PARR
Plantarflexion	41.11	42.24
Dorsiflexion	24.89	25.92
Inversion	16.28	16.46
Eversion	15.80	16.11
Adduction	30.96	33.71
Abduction	28.40	30.49

## Data Availability

All the data used to support the findings of this study are available from the corresponding author upon request.
